# Retrospective Analysis of Infection Factors in Secondary Internal Fixation after External Fixation for Open Fracture of a Long Bone: A Cohort of 117 Patients in a Two-Center Clinical Study

**DOI:** 10.1155/2022/7284068

**Published:** 2022-06-30

**Authors:** Shanwen Zhao, Zelin Ye, Canjun Zeng, Lei Zhang, Juanyu Huang, Wensheng Zhang, Runguang Li

**Affiliations:** ^1^Department of Foot and Ankle Surgery, Center for Orthopaedic Surgery, The Third Affiliated Hospital of Southern Medical University, Guangzhou 510610, China; ^2^Orthopaedic Hospital of Guangdong Province, Guangzhou 510610, China; ^3^Academy of Orthopaedics, Guangzhou, 510610 Guangdong Province, China; ^4^Guangdong Provincial Key Laboratory of Bone and Joint Degenerative Diseases, Guangzhou 510280, China; ^5^Division of Orthopaedics and Traumatology, Department of Orthopaedics, Nanfang Hospital, Southern Medical University, Guangzhou 510515, China; ^6^Department of Spine Surgery, Center for Orthopaedic Surgery, The Third Affiliated Hospital of Southern Medical University, Guangzhou 510610, China

## Abstract

**Purpose:**

To investigate infection risk factors after secondary internal fixation (IF) of open fracture of a long bone with removed fixation frame and explore the safe range of feasible operation for abnormal inflammatory indicators.

**Methods:**

Clinical data of 117 cases of open fracture of a long bone that underwent temporary external fixation (EF) in one stage and IF in two stages were retrospectively analyzed. Collected data included age, sex, Gustilo type, multiple injuries, debridement time, duration of EF, needle infection, interval of conversion to IF after external fixator, preoperative white blood cell (WBC), erythrocyte sedimentation rate (ESR), C-reactive protein (CRP), albumin (ALB), blood glucose, and prognosis. We selected these factors for univariate analysis of postoperative surgical site infection (SSI) and multivariate logistic regression analysis of statistically significant risk factors and created receiver operating characteristic (ROC) curves to compare the diagnostic efficiency of each index and determine the optimal screening point.

**Results:**

We followed up 117 patients, with 130 limbs affected. Univariate analysis showed that ESR, CRP, ALB, WBC, EF time, and Gustilo fracture type were significantly associated with SSI. Multivariate logistic regression analysis showed that CRP, duration of EF, and Gustilo fracture type were independently associated with postoperative infection. Area under ROC curves for WBC, ESR, and CRP were 69.7%, 73.2%, and 81.2%.

**Conclusions:**

We demonstrated the role of Gustilo classification of open fractures in predicting postoperative infection, especially for open fractures above type III. If the inflammatory indexes return to normal or show a downward trend, and the second-stage IF operation is performed within the cutoff values, postoperative recurrent infection was reduced.

## 1. Introduction

Open fractures of long bones of extremities are one of the common diseases in the field of trauma. The treatment of severe open fractures is complex because of the long treatment cycle and high difficulty. When infection occurs, repeated debridement, delayed wound healing, and even amputation are often needed [1–3]. For some patients with open fracture, staging treatment is advocated because of their poor physiological condition or soft tissue state. Initial, rapid, and temporary external fixation (EF) is performed in the early stage, whereas secondary internal fixation (IF) is performed after the general or local soft tissue conditions improve. This approach can improve the survival rate of patients and the success rate of treatment, and it also can reduce the incidence of complications. Therefore, two-stage treatment consisting of temporary fracture EF followed by IF is a safe and effective treatment [4].

The specific timing of the two-stage treatment of open fractures of long bones of extremities and the risk factors of postoperative surgical site infection (SSI) remain controversial [5]. There are a variety of risk factors for postoperative recurrent infection. Among them, a large number of studies have reported that preoperative infection indexes, such as C-reactive protein (CRP) level, erythrocyte sedimentation rate (ESR), and calcitonin (PCT) level, are independent risk factors for postoperative infection. Stucken et al. showed that when the infection indexes, such as white blood cell (WBC) count, ESR, and CRP level, increased, the predictive probability of perioperative infection was 86% [6, 7]. The increase in preoperative inflammatory markers also has been linked to postoperative infection after lumbar surgery [8]. Although a large number of studies have shown that the increase in preoperative inflammatory markers is related to postoperative infection, few studies have further analyzed the safe range of preoperative abnormal inflammatory markers for feasible surgery. In addition, after EF, infection indicators are difficult to be reduced to normal in a short amount of time. Therefore, after comprehensive consideration of patients' situation, some surgeons choose to treat patients with secondary IF, while inflammation indicators are still high and the risk of postoperative infection is unknown [6]. Therefore, it is of great clinical significance to further explore the safe range of preoperative abnormal inflammatory indicators. In addition, consensus still has not been reached on the EF time and conversion interval time in clinical practice [9, 10]. We conducted a retrospective analysis of 117 patients to explore the risk factors of infection after secondary IF of open fractures of long bones with removed fixation frames. Moreover, we analyzed the safe range of abnormal inflammatory biomarkers for feasible surgery.

## 2. Materials and Methods

### 2.1. Research Design and Surgical Methods

This retrospective clinical study was conducted in two grade A tertiary hospitals from January 2017 to May 2020 to track the development of SSI after two-stage treatment of open fractures of long bones of extremities. In this study, two trained investigators extracted data from electronic medical records (EMR) for patients over 15 years old who had undergone open fracture surgery. Personal data, injury mechanism, type of fracture, location of fracture, and severity of soft tissue injury were recorded at admission. After admission, all patients underwent the relevant preoperative examination and were subjected to fluid replacement, as well as antibacterial and anti-inflammatory treatment after definite diagnosis. After preoperative evaluation, one-stage debridement and external fixator installation were performed. After the operation, final IF was performed after the soft tissue condition was stable and the wound surface recovered. Antibiotics were routinely used during the perioperative period, and the wound dressing was changed regularly. According to the postoperative follow-up of the occurrence of infection at the fracture site, the patients were categorized into an infection group and a noninfection group.

### 2.2. Criteria for Inclusion and Exclusion of Cases

The inclusion criteria were as follows: (1) age ≥ 15 years, (2) open fractures of long bones of extremities treated with EF and IF, and (3) postoperative follow − up ≥ 12 months. Case exclusion criteria were as follows: (1) need for long-term bone transport technique because of too many bone defects, (2) systemic connective tissue autoimmune diseases, (3) low immune function, and (4) incomplete follow-up data.

### 2.3. Data Collection and Variable Definition

The study included 20 variables to study the risk factors for SSI after delayed IF. These variables were divided into the following five groups: demographic-related variables, including age, sex, and occupation; variables related to the basic characteristics of fractures, including Gustilo classification of fractures (types I, II, IIIA, IIIB, and IIIC [11]), injury location and comminution degree (AO classification), injury mechanism (car accident, high fall, or other causes), multiple injuries (+ or −), and soft tissue injury (mild, moderate, and severe); perioperative- and operative-related variables, including debridement time (≤6 h or >6 h), fixation method (internal or EF), duration of EF (≤14 d, 14–28 d, or ≥28 d), preoperative albumin (ALB) (35–55 g/L), WBC count (4–10 × 10^9^/L), neutrophil count (1.80–6.30 × 10^9^/L), CRP (0–6 mg/L), ESR (male, 0–15 mm/h; female, 0–20 mm/h), and fasting whole blood glucose (3.9–6.1 mmol/L); postoperative nursing-related variables, including whether there was needle infection before the conversion of IF (+ or −); and prognosis index, that is, whether there was SSI after IF (+ or −). According to the degree of infection and the mode of treatment, the infection was classified into one of the following three grades: grade 1 (mild infection), which could be improved by conservative treatment; grade 2 (moderate infection), which needed debridement surgery; and grade 3 (severe infection), requiring complete debridement after removal of IF or osteotomy after focus debridement. If there were different degrees of infection during the follow-up period, we chose the highest level for inclusion in in this study [12].

### 2.4. Data Analysis

To account for the missing values in some variables, we eliminated outliers and took the average to replace the missing values. Frequencies and percentages were used to describe classified variables. For the univariate analysis of classification covariates, we used the chi-square test or Fisher exact probability test. The risk factors related to SSI after delayed IF in the univariate analysis were input into multivariate logistic regression analysis to determine the independent predictors of postoperative infection. Logistic regression analysis used step-by-step backward elimination method to exclude mixed covariates from the multivariate model. *P* < 0.05 was considered statistically significant. Finally, the Hosmer–Lemeshow test was used to evaluate the goodness of fit of the final model, with *P* > 0.05 as an acceptable degree of fit. Finally, we created receiver operating characteristic (ROC) curves of the statistically significant indicators, used the area under the ROC curve (AUC) [13–15] to evaluate the diagnostic efficiency of the index, and determined the cutoff point [16]. *P* < 0.05 was considered statistically significant. SPSS22.0 statistical software was used for data analysis.

## 3. Results

A total of 117 patients were included in the study, including 88 males (75.2%) and 29 females (24.8%). Among them, 13 patients had two open fractures at the same time, and both fractures were treated with delayed IF. To facilitate the statistical analysis of data, we assumed that a total of 130 patients were included. In our retrospective study, after the treatment of open fracture of long bones with an external fixator and IF, 17 cases received the diagnosis of SSI, with the postoperative infection rate of 13.08%. No infection was found in 113 cases.

### 3.1. Results of the Univariate Analysis for Each Variable

We did not find a significant association between SSI and age, sex, fracture AO classification, fracture location, multiple injuries, debridement time, neutrophil count, blood glucose level, and needle tract infection (*P* > 0.05). The results showed that Gustilo classification (*P* = 0.001), duration of EF (*P* = 0.031), WBC count (*P* = 0.044), CRP level (*P* = 0.012), ESR (*P* = 0.031), and ALB level (*P* = 0.019) were important factors affecting the occurrence of SSI. The results of the univariate analysis are given in Table 1.

### 3.2. Results of the Multivariate Logistic Regression Analysis

Multivariate logistic regression analysis included Gustilo classification, EF time, WBC count, CRP level, ESR, and ALB level. The results showed that CRP level (odds ratio [OR] = 38.002; 95% CI, 3.718–388.390; *P* = 0.002), Gustilo classification (*P* = 0.018), and EF time (*P* = 0.026) were independently associated with SSI after operation. Gustilo classification of fracture was the most significant predictor of postoperative recurrent infection. Analysis of subvariables of Gustilo fracture classification showed the following results: type IIIA (OR = 1.030; 95% CI, 0.138–7.688; *P* = 0.977), type IIIB (OR = 4.052; 95% CI, 0.631–26.017; *P* = 0.14), and type IIIC (OR = 16.845; 95% CI, 1.987–142.816; *P* = 0.01).

The analysis of the subvariables of the duration of EF showed the following results: 14–28 days (OR = 2.096; 95% CI, 0.294–14.939; *P* = 0.460) and ≥28 days (OR = 7.837; 95% CI, 1.706–36.006; *P* = 0.008). The results of the Hosmer–Lemeshow test showed that the goodness of fit was good (*P* = 0.835). The results of the multivariate logistic regression analysis are given in Table 2.

### 3.3. ROC Curves of WBC Count, ESR, and CRP Level

The diagnostic efficiency of WBC count, ESR, and CRP level was analyzed by drawing ROC curves. As shown in the figures, the AUCs of WBC, ESR, and CRP were 69.7%, 73.2%, and 81.2%, respectively, and the best cutoff values were 6.69 × 10^9^/L, 39.45 mm/1 h, and 18.79 mg/L, respectively (Figure 1). The results showed that the diagnostic efficiency of CRP level was the highest among the three, and the sensitivity of WBC count was high, but its specificity was low. The sensitivity of ESR was low, but its specificity was high (Table 3).

## 4. Discussion

The two-stage treatment of open fractures is controversial, mainly because the factors of infection are not clear [17]. In this study, six risk factors associated with SSI were identified by the univariate analysis, including Gustilo classification of fracture, EF time, WBC count, CRP level, ESR, and ALB level. Through the multivariate logistic regression analysis, we showed that CRP level, Gustilo fracture classification, and EF time were independently associated with SSI. Among the mentioned predictors, five risk factors were modifiable, and we observed that they played an important predictive role in protecting patients from postoperative infection.

We found that infection indexes, such as WBC count, ESR, and CRP level, were independent risk factors for SSI; further analyzed by ROC curves, their best cutoff values were 6.69 × 10^9^/L, 39.45 mm/1 h, and 18.79 mg/L, respectively. According to the results of our analysis, the risk of postoperative SSI can be reduced by controlling the preoperative abnormal inflammation indexes within the optimal cutoff value before operation. Hardcastle et al. [18] reported that the abnormal increase in ESR or CRP level before operation increased the possibility of infection and reoperation after total knee arthroplasty. The increases in ESR and CRP were important risk factors for postoperative infection, and the time of CRP reaction was related to the time of treatment. CRP level usually reached its peak 2 days after admission or operation, and then, it decreased. During the decline, if the CRP level increased again, it indicated that the patient was at a risk of infection [19, 20]. In addition, many reports have shown that WBC count, CRP level, ESR, and PCT level play an important role in the diagnosis of early infection [7, 21].

As far as we know, however, although many studies have shown that the increase in preoperative inflammatory indexes is related to postoperative infection, few studies have analyzed the safe range of preoperative abnormal inflammatory indexes. In this context, we identified the risk factors for SSI after secondary IF and further analyzed the safe range of preoperative abnormal inflammation indexes for feasible operation to provide a basis for clinicians to evaluate the risk of SSI after secondary IF. In addition, although preoperative ESR and CRP level are effective screening methods, occult infection may still be missed. In short, when preoperative ESR and CRP level are abnormally elevated, their diagnostic value is limited [22]. The value of PCT combined with CRP in the detection of early postoperative infection is higher than that of CRP when tested alone [23]. Therefore, we can use CRP and ESR combined with PCT to improve the diagnostic sensitivity for infection after IF. However, because some patients in this study did not carry out PCT test, we did not further study the role of PCT. In further work, we plan to add PCT test.

Through the univariate analysis by the chi-square and Fisher tests, we showed that a low ALB level was one of the risk factors for postoperative infection. Kamath et al. [24] reported the relationship between malnutrition and postoperative complications of total knee arthroplasty. Thus, preoperative hypoalbuminemia could be used as a potential preoperative predictor of prognosis. In addition, a significant difference has been reported in 30-day postoperative complications between patients with a normal preoperative ALB level and those with a low ALB level after initial total joint replacement or revision [25]. A hypothetical reason for the increased incidence of adverse outcomes after surgery is that malnutrition caused by low ALB levels affect wound healing because of decreased collagen synthesis and fibroblast proliferation. Another possible explanation for the importance of ALB is that hypoalbuminemia reduces the inflammatory response that usually protects against infection, while the complete innate and adaptive immune responses depend on ALB. ALB plays an important role in antibacterial defense and repair [25, 26]. Therefore, it is essential to assess in advance the risk of postoperative infection resulting from low ALB levels and to treat patients with low ALB both preoperatively and perioperatively.

Gustilo classification of open fractures was the most significant predictor of SSI [27]. The logistic regression analysis showed that Gustilo classification was an independent risk factor for SSI (*P* = 0.018); the analysis of the subvariables of Gustilo classification showed the ORs of 1.030, 4.052, and 16.845 for types IIIA, IIIB, and IIIC, respectively. Hence, higher Gustilo type is associated with higher risk of SSI; for example, for type IIIC fractures, the risk of infection is 16.8 times higher than that for type I and II fractures. Thakore et al. [27] reported that Gustilo classification of open tibial fractures was by far the strongest predictor of nonunion and infection. Gustilo classification is often used by surgeons as an indicator of injury severity and a prognostic tool. Therefore, patients with high-grade Gustilo open fractures should be monitored more closely, and more active treatment programs should be taken from preoperative to postoperative period to prevent the occurrence of SSI.

Regarding the fixed time and conversion interval time of the external frame, the results of this study showed that with the extension of the carrying time of the temporary external fixator, especially if external fixator time was more than 28 days, the postoperative infection rate showed an overall upward trend. We did not find a significant association between the occurrence of SSI and the interval time of conversion to IF after external fixator installation. At present, consensus still has not been reached on the optimal time for changing EF to IF. Bhandari et al. [10] found that the infection rate increased when duration of EF was more than 28 days and the interval of secondary conversion was more than 14 days. Therefore, they suggested that the duration time of the external fixator should not exceed 28 days and that the interval of IF of secondary conversion should not exceed 14 days. Some scholars believe that when the temporary external fixator is retained for 5–10 days, when the patient's general condition or local soft tissue improves, the temporary external fixator can be converted into deterministic IF [28, 29]. However, Rixen et al. [9] found that after short-term EF, the best conversion results were obtained when the conversion interval was more than one week (at least 9 days). In that context, although our research results did not suggest that a correlation exists between the conversion interval and SSI, we cannot completely ignore its importance. To establish a clear scheme of secondary IF for the treatment of open long bone fractures, a prospective randomized study is needed.

This study had several limitations. First, in terms of research methods, this study was a retrospective study, which reduced the credibility of the evidence to a certain extent. In addition, in terms of data processing, because the cases were collected in two different hospitals, the detection time of each patient's preoperative inflammation indexes was not uniform, and the preoperative test results of some patients were incomplete. The processing method that we adopted was to eliminate outliers and take the average to replace the missing values, so the analyzed data have a certain error.

In addition, according to the reports in the literature, many other factors affect postoperative infection, such as preoperative use of antibiotics, wound closure time, operation time, osteofascial compartment syndrome, and smoking [30–33]. These factors were not considered in our study. Therefore, we plan to collect and analyze other related factors in further work.

## 5. Conclusions

We proved once again that Gustilo classification of open fractures can predict postoperative infection, especially for open fractures above type III. When the indexes of WBC, CRP, and ESR returned to normal or the abnormal inflammatory indexes were controlled within the optimal cutoff value, the occurrence of postoperative infection could be reduced.

## Figures and Tables

**Figure 1:** (a) Plots of WBC levels in SSI and NO SSI groups. (b) ROCs of WBC for SSI diagnosis. *P* < 0.05 was considered statistically significant. (c) Plots of ESR levels in SSI and NO SSI groups. (d) ROCs of ESR for SSI diagnosis. *P* < 0.05 was considered statistically significant. (e) Plots of CRP levels in SSI and NO SSI groups. (f) ROCs of CRP for SSI diagnosis. *P* < 0.05 was considered statistically significant.

**Table 1:** Univariate predictors for SSI of preoperative variables.

Variable	SSI (*N* = 17)	No SSI (*N* = 113)	Infection rates (%)	*P* value
Age (years)				
≤50 years	14 (82.4%)	87 (77.0%)	14/101 (13.9%)	0.762
>50 years	3 (17.6%)	26 (23.0%)	3/29 (10.3%)	
Gender, number (%)				
Male	15 (88.2%)	85 (75.2%)	15/100 (15%)	0.357
Female	2 (11.8%)	28 (24.8%)	2/30 (6.7%)	
Injured area				
Humerus	0	5 (4.4%)	0	0.416
Ulna and radius	1 (5.9%)	15 (13.3%)	1/16 (6.3%)	
Femoral	4 (23.5%)	24 (21.2%)	4/28 (14.3%)	
Tibia and fibula	12 (70.6%)	69 (61.1%)	12/81 (14.8%)	
Multiple trauma				
+	15 (88.2%)	78 (69.0%)	15/93 (16.1%)	0.149
-	2 (11.8%)	35 (31.0%)	2/37 (5.4%)	
Type of open fracture (Gustilo classification)				
I or II	2 (11.8%)	46 (40.7%)	2/48 (4.2%)	0.001^a^
IIIA	3 (17.7%)	36 (31.9%)	3/39 (7.7%)	
IIIB	6 (35.3%)	23 (20.4%)	6/29 (20.7%)	
IIIC	6 (35.3%)	8 (7.1%)	6/14 (42.8%)	
AO type				
A	3 (17.6%)	39 (34.5%)	3/42 (7.1%)	0.416
B	6 (35.3%)	32 (28.3%)	6/38 (15.8%)	
C	8 (47.1%)	42 (37.2%)	8/50 (16.0%)	
Degree of soft tissue damage				
Mild	10 (58.8%)	69 (61.1%)	10/79 (12.7%)	0.176
Moderate	1 (5.9%)	23 (20.3%)	1/24 (4.2%)	
Severe	6 (35.3%)	21 (18.6%)	6/27 (22.2%)	
Debridement time				
≤6 h	5 (29.4%)	26 (23.0%)	5/31 (16.1%)	0.296
>6 h	12 (70.6%)	87 (77.0%)	12/99 (12.1%)	
Duration of external fixation				
≤14 d	4 (23.5%)	58 (51.3%)	4/62 (6.5%)	0.031^a^
14-28 d	2 (11.8%)	19 (16.8%)	2/21 (9.5%)	
≥28 d	11 (64.7%)	36 (31.9%)	11/47 (23.4%)	
Pin-site infection				
+	4 (23.5%)	8 (7.1%)	4/12 (33.3%)	0.052
-	13 (76.5%)	105 (92.9%)	13/118 (11.0%)	
WBC (4 − 10 × 10^9^/L)				
4 − 10 × 10^9^/L	10 (58.8%)	94 (83.2%)	10/104 (9.6%)	0.044^a^
>10 × 10^9^/L	7 (41.2%)	19 (16.8%)	7/26 (26.9%)	
*N* (1.80 − 6.30 × 10^9^/L)				
1.80 − 6.30 × 10^9^/L	15 (88.2%)	92 (81.4%)	15/107 (14.0%)	0.736
>6.30 × 10^9^/L	2 (11.8%)	21 (18.6%)	2/23 (8.7%)	
CRP (0-6 mg/L)				
≤6 mg/L	3 (17.6%)	41 (36.3%)	3/44 (6.8%)	0.012^a^
>6 mg/L	14 (82.4%)	72 (63.7%)	14/86 (16.3%)	
ESR (male 0-15 mm/h, female 0-20 mm/h)				
≤15/20 mm/h	2 (11.8%)	41 (36.3%)	2/43 (4.7%)	0.031^a^
>15/20 mm/h	15 (88.2%)	72 (63.7%)	15/87 (17.2%)	
Fasting plasma glucose (3.9-6.1 mmol/L)				
3.9-6.1 mmol/L	15 (88.2%)	94 (83.2%)	15/109 (13.8%)	0.862
>6.1 mmol/L	2 (11.8%)	19 (16.8%)	2/21 (9.5%)	
ALB (35-55 g/L)				
<35 g/L	9 (52.9%)	27 (23.9%)	9/36 (25.0%)	0.019^a^
35-55 g/L	8 (47.1%)	86 (76.1%)	8/94 (8.5%)	

^a^ *P* < 0.05 denotes significance.

**Table 2:** Variables tested for multivariate analysis.

Variables	*P* value	S E	Wald	OR	95% CI	Hosmer and Lemeshow test
CRP	0.002^a^	1.186	9.409	38.002	3.718-388.390	
Type of open fracture (Gustilo classification)	0.018^a^		10.044			0.835
IIIA	0.977	1.025	0.001	1.030	0.138-7.688	
IIIB	0.140	0.949	2.175	4.052	0.631-26.017	
IIIC	0.01^a^	1.091	6.706	16.845	1.987-142.816	
Duration of external fixation	0.026^a^		7.282			
14-28 d	0.460	1.002	0.545	2.096	0.294-14.939	
≥28 d	0.008^a^	0.778	7.003	7.837	1.706-36.006	

CI: confidential interval. ^a^*P* < 0.05 denotes significance. Hosmer and Lemeshow test: *P* > 0.05 denotes that the goodness of fit is acceptable.

**Table 3:** Discriminatory strengths of the three inflammatory biomarkers.

Infection markers	AUC	95% CI	Optimal cutoff value∗	Sensitivity	Specificity
WBC (×10^9^/L)	0.697	0.572-0.821	6.69	94.1%	38.7%
ESR (mm/1 h)	0.732	0.608-0.856	39.45	58.8%	85.8%
CRP (mg/L)	0.812	0.698-0.926	18.79	82.4%	79.6%

∗The optimal cutoff value was obtained by calculating the maximum Youden index (sensitivity + specificity–1).

## Data Availability

The data used to support the findings of this study are included within the article.
